The article "The association between HIV tri-therapy with the development of Type-2 Diabetes Mellitus in a rural South African District: A case-control study" was published in 2020. Journal: PLoS One.

# The association between HIV tri-therapy with the development of Type-2 Diabetes Mellitus in a rural South African District: A case-control study

**DOI:** 10.1371/journal.pone.0244067

**Published:** 2020-12-31

**Authors:** Nokwanda E. Bam, Sikhumbuzo A. Mabunda, Jafta Ntsaba, Teke Apalata, Sibusiso C. Nomatshila, Wezile Chitha

**Affiliations:** 1 Department of Nursing, Walter Sisulu University, Mthatha, South Africa; 2 The George Institute for Global Health, University of New South Wales, Sydney, Australia; 3 Department of Laboratory Medicine, Walter Sisulu University, Mthatha, South Africa; 4 Department of Public Health, Walter Sisulu University, Mthatha, South Africa; 5 Health Systems Enablement & Innovation Unit, University of the Witwatersrand, Johannesburg, South Africa; University of Sassari, ITALY

## Abstract

**Background:**

Combination antiretroviral drugs (cARVs) prolong patients’ lives but are unfortunately thought to increase complications related to metabolic disorders including type-2 Diabetes Mellitus (DM). We sought to confirm the association of cARVs with type-2 DM and ascertain the extent of this association in a rural South African setting.

**Methods:**

A case-control study of 177 (33.33%) cases with HIV/AIDS and type-2 DM were selected and compared with 354 (66.67%) non-DM HIV/AIDS unmatched controls from a rural district of South Africa’s third most populous province (Eastern Cape). Cases were identified from community health centres using the district health information system, and controls were identified using simple random sampling from the same health facilities. Odds Ratios (OR), together with 95% confidence intervals, were calculated for all the univariable and multivariable logistic analyses.

**Results:**

This study found that cARVs significantly increased the occurrence of type-2 DM among HIV patients. Patients on protease inhibitors (PIs) were at least 21 times significantly (p<0.0001) more likely to be diabetic than those on the fixed dose combination (FDC); those on stavudine (D4T) and zidovudine (AZT) were 2.45 times and 9.44 times respectively more likely to be diabetic than those on FDC (p<0.05). The odds of diabetes increased by more than three-folds for those who had been on antiretroviral drugs for more than 6 years (p<0.005).

**Conclusion:**

This study has been able to establish the association between cARVs and type-2 DM. It therefore proposes consideration of the usage of AZT, D4T, lopivavir and ritonavir for the treatment of HIV. The study further proposes more prospective research to test these findings further.

## Introduction

Tri-therapy or combination antiretroviral therapies (cARVs) have improved the life-course of HIV/AIDS from an acute killer disease to a chronic manageable disease [1]. This can be largely attributed to the huge progress antiretroviral drugs (ARVs) have made in improving adherence and the immune system’s response of the people living with HIV/AIDS (PLWHIV), thus increasing their life expectancy [2, 3]. Some scholars postulate that the quality of life among PLWHIV would be much better if these drugs were not associated with metabolic illnesses and risks including type-2 diabetes mellitus (DM), insulin resistance, lipodystrophy and dyslipidaemia [4–6].

These metabolic risks are thought to be associated with the duration of exposure to cARVs [6]. Insulin resistance and/or the factors related to disturbance in glucose metabolism especially dyslipidaemia has the potential to threaten the quality of life and wellness of patients as they escalate inflammation and the onset of diabetes mellitus [7]. Specific characteristics of HIV related lipodystrophy are noted by lipo-atrophy on the face, buttocks and abdomen due to nucleoside/nucleotide reverse transcriptase inhibitors (NRTIs) and lipo-hypertrophy possibly linked to protease inhibitors (PIs) [6].

Since 2013, South Africa has advanced to the use of a fixed drug/dose combination (FDC) made up of tenofovir (TDF), emtricitabine (FTC) and efavirenz (EFV) as a first line drug for the treatment of HIV [8, 9]. In March 2020, the guidelines were updated to have a FDC of TDF, lamivudine (3TC) and Dolutegravir (an integrase inhibitor) as a first line drug for non-pregnant (or planning to conceive) patients older than 10-years and weighting more than 35-kg [10]. The TDF, 3TC and Dolutegravir regimen (TLD) [10] will take a while to be transitioned throughout the country. In addition, there are still some patients on historical regimen consisting of combination drugs made up either of two NRTIs (zidovudine (AZT) or stavudine (D4T) and 3TC) and a non-nucleoside reverse transcriptase inhibitors (NNRTI = nevirapine or efavirenz). Sometimes the NNRTI is replaced with a PI (lopinavir (LPV) or ritonavir (RTV) [8, 9].

Hall et al. previously warned about high increases in the incidence and prevalence of type-2 diabetes in sub-Saharan Africa (SSA) due to urbanisation, improved food access and modern living [11]. Moleutze et al. previously projected an increase in the DM burden for South Africa that was independent of the HIV/AIDS burden [12]. Furthermore, a multi-morbidity situation co-exists; the number of people living with both HIV/AIDS and Diabetes in SSA is increasing [3]; and yet very little research has been done on the association of diabetes mellitus and cARVs in a rural South African population [2].

## Methods

### Participants and recruitment

This study was conducted in primary care facilities of the OR Tambo District in South Africa’s Eastern Cape Province. This is the second biggest province by surface area and the third most populous [13]. It has eight (8) health Districts, OR Tambo District being the largest was conveniently chosen for this study [13]. The study site included ten (10) community health centres (CHCs) and 140 clinics.

A quantitative case-control study design was used to compare HIV positive patients who were on cARVs with HIV positive patients who were on non-combined antiretroviral therapy to assess their odds of developing type-2 DM. Cases were therefore defined as type-2 DM patients on treatment with comorbid HIV and on antiretroviral therapy (whether combined or not). Controls were HIV positive patients on antiretroviral therapy (whether combined or not) who did not have a DM diagnosis (whether type-1 or type-2).

Cases (DM patients) and controls (non-DM patients) were recruited from the same clinics and CHCs of the OR Tambo District at a ratio of 1:2 cases to controls respectively. Cases were extracted from the District Health Information System (DHIS) and invited to participate through their local primary care facilities. DHIS data extracted used the reporting period of 01 April 2015 to 31 March 2016. The aim was to extract all identified cases since comorbid HIV and Diabetes is moderately rare. Simple random sampling was used to select two controls per case in each of the five sub-districts daily until the required sample size was reached.

Participants were sourced from two (2/10) CHCs and six clinics (6/140). Only data from participants who met the inclusion criteria were considered; that is, adult patients older than 18 years who were on ARVs for at-least a year and patients with type-2 DM on treatment for cases. We excluded HIV negative patients; patients with type 1 DM and gestational DM and those who were less than 20 years of age.

### Measures

Information was sourced using a structured self-administered questionnaire (annexure A) adapted for HIV from the World Health Organization Stepwise tool for chronic diseases [14] translated from English to the local language (isiXhosa) and distributed to participants who signed the consent to participate. This validated questionnaire collected information on demographic characteristics and medical history. The principal investigator measured the height in centimetres, weight in kilograms, and upper arm blood pressure using a digital stadiometer (seca 787) and a digital blood pressure monitor (Omron HEM-7321-E) respectively. The instruments were piloted on three participants attending primary care in one of the communities prior to commencement of the study. Information emerging from pre-testing the tools enhanced and modified the data collection instruments. Medical records were used for clinical measurements and confirmation of participants’ clinical records.

### Analysis

Microsoft Excel 2016 (Microsoft Corporation, Seattle, USA) was used to capture data and STATA version 14.1 (Stata Corp LP, College Station, Texas, USA) was used for data management and analysis. Selected predictors included HIV parameters: CD4 count, viral load & ARVs) were analysed to seek the associations of type-2 diabetes mellitus in HIV/AIDS patients. Descriptive statistics and frequency distributions were analysed through medians, interquartile range (IQR) and proportions. Categorical variables were described using frequency tables and percentages whereas continuous data were explored for normality using the Shapiro Wilk test. The Wilcoxon sum rank test was used to compare the differences between two medians. The two-sample test of proportions was used to compare two proportions of cases and controls. Odds Ratios (OR), together with 95% confidence intervals (95% CI), were calculated for all the univariable and multivariable logistic analyses. Purposeful selection of variables [15] was undertaken to determine the best fitting model to be included in the multivariable model. A p-value of 0.05 or less was considered a statistically significant result.

### Ethical approval and consent to participate

Formal ethical approval was sought and obtained from the Research Ethics Committee of Walter Sisulu University (HREC number: 075/2016). Gatekeeper permission to conduct the research (patient interviews and health information system access) was obtained from the Eastern Cape Department of Health Provincial Health Research Committee (approval number: EC_2016RP21_875) and OR Tambo District and sub-districts health management. Research participants were informed about the purpose and objectives of the study prior to obtaining voluntary, written informed consent for participation in the study.

## Results

Summary demographic and clinical characteristics of participants are presented in Table 1. Of all the participants, 33.33% (177/531) were cases and 66.67% (354/531) were controls. Almost 90% were female (463/531 or 87.19%) who were mostly (296/531 or 55.74%) below the age of 40 years. Cases had been on ARVs for 2 years longer (median = 6 years; IQR = 3–8 years) than controls (median = 4 years; IQR = 2–7 years) and this was statistically significant (p<0.0001) (Fig 1). In addition, there were significantly more controls (58.19%) than cases (42.37%) who had been on ARVs for between 2 and 5 years (p = 0.001). All participants who were not on FDC received lamivudine (n = 172 or 32.39%). AZT and D4T were used by 114 (21.47%) and 10.92% (58/531) of participants respectively. Only 10.17% of participants (54/531) were on PIs (LPV = 31, RTV = 23). The balance of patients, 118 or 22.22% were on NNRTIs (EFV = 116 and NVP = 2).

**Fig 1:** Duration (years) on ARVs for cases and controls.

**Table 1:** Summary characteristics of cases and controls.

Demographics characteristics (N = 531)	Cases		Controls		p-value
	Diabetic		Non-Diabetic		
Sex; n (%)					
Female	154	(87.01)	309	(87.29)	0.927
Male	23	(12.99)	45	(12.71)	0.927
BMI, kg/m^2^; Median (IQR)	25	(23–29)	25	(23–29)	0.290
Age, years; Median (IQR)	37	(31–46)	38	(31–46)	0.882
Age, years; n (%)					
<40	100	(56.50)	196	(55.37)	0.805
≥40	77	(43.50)	158	(44.63)	0.805
ART regimen; n (%)*					
Fixed dose combination	69	(38.98)	290	(81.92)	<0.0001
D4T/3TC/EFV	21	(11.86)	37	(10.45)	0.623
AZT/3TC/EFV	40	(22.60)	18	(5.08	<0.0001
AZT/3TC/LPV	27	(15.25)	4	(1.13)	<0.0001
AZT/3TC/RTV	19	(10.73)	4	(1.13)	<0.0001
AZT/3TC/NVP	1	(0.56)	1	(0.56)	0.616
CD4+ cell count, g/dL; Median (IQR)	550	(370–750)	499	(360–714)	0.176
CD4 level, g/dL; n (%)					
<200	21	(11.86)	35	(9.89)	0.484
200–499	52	(29.38)	143	(40.40)	0.013
≥500	104	(58.76)	176	(49.72)	0.049
Viral load, copies/mL; Median (IQR)	0	(0–20)	0	(0–20)_	0.646
Viral load, copies/mL; n (%)					
Lower than detectable	128	(72.32)	257	(72.60)	0.945
1–100	26	(14.69)	64	(18.08)	0.326
101–10 000	23	(12.99)	33	(9.32)	0.194
Years on ARVs; n (%)**					
≤1	7	(3.95)	30	(8.47)	0.054
2–5	75	(42.37)	206	(58.19)	0.001
6–10	87	(49.15)	110	(31.07)	<0.0001
>10	8	(4.52)	8	(2.26)	0.151
ARV complications; n (%)					
Yes	23	(12.99)	15	(4.24)	0.0002
No	154	(87.01)	339	(95.76)	0.0002

*3TC = lamivudine; AZT = zidovudine; D4T = stavudine; EFV = efavirenz; LPV = lopinavir; NVP = nevirapine; RTV = ritonavir.

**Years on ARVs refers to the duration of initiation on ARVs but not necessarily the duration on the current regimen.

Table 1 further shows that the fixed dose combination was the most used drug for both cases and controls (p<0.0001). There were no statistical differences between those who were on the D4T/3TC/EFV (p = 0.623) and AZT/3TC/NVP (p = 0.616) when comparing cases and controls. However, there were proportionally more cases than controls on AZT/3TC/EFV (p<0.0001), AZT/3TC/LPV (p<0.0001) and AZT/3TC/RTV (p<0.0001). Significantly more controls (95.76% or n = 339) than cases (87.01% or n = 154) reported ARV related complications (p-value = 0.0002).

Table 2 depicts the univariable analysis and their association with type-2 DM. Cases were three times significantly more likely to report complications related to ARVs compared to non-diabetic participants (OR = 3.38; CI: 1.71–6.65; p-value <0.0001).

**Table 2:** Univariable analysis of patients’ demographic characteristics and determinants of type-2 diabetes mellitus.

Characteristic	n	(%)	OR	(95% Confidence Interval)	p-value
	N = 531				
**Sex**					
** Females**	154/463	(33.26)	ref		1
** Males**	23/68	(33.82)	1.03	(0.60–1.76)	0.927
BMI, kg/m^2^					
** ≤25**	93/297	(33.31)	ref		1
** 26–29**	42/111	(37.84)	1.34	(0.85–2.11)	0.213
** ≥30**	42/123	(34.15)	1.14	(0.73–1.78)	0.557
**Age, years**					
** <40**	100/296	(33.78)	ref		1
** ≥40**	77/235	(32.77)	1.05	(0.73–1.51)	0.805
**CD4 level g/dL**					
** 200–499**	52/195	(26.67)	ref		1
** <200**	21/56	(37.50)	1.65	(0.88–3.09)	0.118
** ≥500**	104/280	(37.14)	1.63	(1.09–2.42)	0.017
**Viral load**					
^#^LDL	128/385	(33.25)	ref		1
** 1–100**	26/90	(28.89)	0.82	(0.49–1.35)	0.131
** >100**	23/56	(41.07)	1.40	(0.79–2.48)	0.250
**ARV complications**					
** No**	154/493	(31.24)	ref		1
** Yes**	23/38	(60.53)	3.38	(1.71–6.65)	<0.0001
**Years on ARV**					
** ≤1**	7/37	(18.92)	ref		1
** 2–5**	75/281	(26.69)	1.56	(0.66–3.70)	0.313
** 6–10**	87/197	(44.16)	3.39	(1.42–8.09)	0.006
** >10**	8/16	(50.00)	4.29	(1.19–15.41)	0.026
**Drug Regimen**					
2 arto^$^	2/295	(0.68)	ref		1
1 arto**	175/236	(74.15)	420.29	(101.50–1740.23)	<0.0001
**ART regimen**					
** FDC**	69/359	(19.22)	ref		1
** D4T/3TC/EFV**	21/58	(36.21)	2.39	(1.31–4.33)	0.004
** AZT/3TC/EFV**	40/58	(68.97)	9.34	(5.05–17.28)	<0.0001
** AZT/3TC/LPv**	27/31	(87.10)	28.37	(9.61–83.74)	<0.0001
** AZT/3TC/RTV**	19/23	(82.61)	19.96	(6.58–60.56)	<0.0001
** AZT/3TC/NVP**	1/2	(50.00)	4.20	(0.26–68.03)	0.312

^#^LDL = Lower than detectable

** 1-art0 = Only on ART

^$^ 2-arto = On ART and at least one other chronic medication.

Whereas the diabetes diagnosis of most cases (61.02% or 108/177) was made whilst they were already on ARVs, 39% of participants were already on DM medication before being initiated on ARVs. The longer the respondents were on ARVs the higher their odds of developing type-2 DM (Table 2). The odds of being Diabetic were four and three times significantly more likely for those on ARVs for more than 10-years (p = 0.026) or 6 to 10 years (p = 0.006) respectively compared to those who had only been on ARVs for not longer than a year.

As compared to HIV infected patients who received the single FDC therapy, all other types of cARVs were associated with higher odds of being diabetic and most were statistically significant except for the 2 outlier participants who received the AZT, 3TC and NVP combination (p = 0.312). There was no statistical difference between the median duration on ARVs between cases and controls (Table 3).

**Table 3:** Median duration on ARV class in years between cases and controls.

ARV Combinations	Cases		Controls		p-value
	Median (IQR): Years				
**Fixed dose combination**	3	(3)	4	(3)	0.212
**D4T/3TC/EFV**	8	(4)	7	(2)	0.400
**AZT/3TC/EFV**	7	(4)	6.5	(3)	0.741
**AZT/3TC/LPV**	8	(3)	6	(3)	0.055
**AZT/3TC/RTV**	8	(4)	7	(1.5)	0.269
**AZT/3TC/NVP**	7	(0)	7	(0)	-

***IQR = Interquartile Range (75^th^ percentile minus 25^th^ percentile).

Table 4 shows the multivariable logistic regression model after controlling for potentials confounders. The ARV regimen was significantly and independently associated with type-2 DM. Except for the AZT/3TC/NVP regimen, all combinations were associated with significantly higher odds (p<0.005) of diabetes mellitus than those on FDC.

**Table 4:** Multivariable logistic analysis.

Characteristic	OR	(95% Confidence interval)	p-value
**Sex**			
** Male**	ref		1
** Female**	1.21	(0.62–2.36)	0.568
**Age, years**			
** ≥40**	ref		1
** <40**	1.30	(0.84–2.01)	0.234
**ART Regimen**			
** Fixed dose combination**	ref		1
** D4T/3TC/EFV**	2.45	(1.35–4.47)	0.003
** AZT/3TC/EFV**	9.44	(5.09–17.51)	<0.0001
** AZT/3TC/LPV**	31.20	(10.41–93.55)	<0.0001
** AZT/3TC/RTV**	21.19	(6.92–64.81)	<0.0001
** AZT/3TC/NVP**	4.23	(0.26–69.00)	0.311

## Discussion

South Africa has the highest HIV prevalence of any nation and has the biggest ARV program globally, accounting for at least 17% of the world’s HIV population [16, 17]. This study aimed to determine the determinants of diabetes mellitus in the HIV/AIDS population in rural South Africa. Even though several studies have been done to assess the association of cARVs with the onset of type-2 DM, a few have been conducted in a rural population [18–20].

This case-control study has been able to identify the association of HIV and type-2 DM in a low-and middle- income country (LMIC) setting. It was able to show increasing odds of diabetes with an increasing duration on cARVs. In addition, for 61% (n = 108) of cases the antiretroviral therapy preceded the type-2 diabetes mellitus diagnosis. Four of the five cARVs were significantly associated with higher odds of type-2 diabetes mellitus when compared to FDC. The only drug combination without a statistically significant association was AZT/3TC/NVP most likely due to its small sample size (n = 2). This study is therefore significant in not only adding to the existing literature but will help improve; quality of care, policy and health service planning, to prevent against the increasing burden of type-2 DM.

This study is consistent with existing literature confirming the association between cARVs and an increase in the prevalence of type-2 DM [18, 21, 22]. For example, among Cameroonians on cARVs, type-2 DM was higher by 31% as opposed to 17% of those who were not on cARVs [18]. In the USA, type-2 DM ranges between 3.8% and 5.8% among HIV positive adults compared to the general population of adults [21]. The odds of diabetes ranged from 2.45 (p = 0.003) when on a stavudine based NRTI and Efavirenz (NNRTI), to 9.44 (p<0.0001) when the D4T was replaced with AZT. This increased even further when the Efavirenz was replaced with either ritonavir (OR = 21.19; p<0.0001) or lopinavir (OR = 31.20; p<0.0001). Patients on AZT or D4T have been previously reported to have an 11.2% and 1.2% respectively higher risk of type-2 DM than general adults in the population [21, 22].

However, the findings of a higher association between type-2 DM and protease inhibitors (lopinavir and ritonavir) are contrary to systematic review findings by Echecopar-Sabogal et al. [19], who did not find an association [19]. The authors did however, find an association between protease inhibitors and metabolic syndrome (a precursor of DM), suggesting the need for follow-up studies of a longer duration [19], which have been strengthened by this retrospective study. A Cameroonian study also failed to find an association between type-2 DM and the AZT/3TC/NVP regimen [18], even though consistent with this study’s findings, the fact that it was only one case and one control makes it impossible to conclude based on that.

The fact that cases were three times significantly more likely to report ARV related complications than controls (p<0.0001), does suggest that DM is one of the major complications for patients on cARVs. Cases were at least 3-times more likely to have been on cARVs compared to controls (p<0.05), further supporting the association of DM with the duration on ARVs. Even though a Cameroonian study did not find effects on glucose metabolism/insulin sensitivity and the ARV duration [20], another study in the same country [18] found an association between type-2 DM and the mean duration on ARVs of 58.6±28.5 months, which is consistent with this study’s findings.

To the knowledge of the researchers, this is the only study that has clearly shown the association of type-2 DM with cARVs through a case-control study. Despite the recent introduction of TLD [10], FDC remains the first line ARV regimen in this setting [8, 9], efforts must therefore be taken to change all those not contra-indicated who are on any other regimen. The use of AZT, D4T, Lopinavir and Ritonavir should be reserved for those patients who have failed all other regimens. Safer NRTIs (Abacavir (ABC)) and protease inhibitors (Darunavir (DRV) and Atazanavir (ATV)) should instead be used in their place as alternative or second line drugs if FDC is contraindicated or failing to suppress the virus.

Even though minimised, the study had some limitations. Firstly, the use of a case-control study meant that researchers relied only on the drug regimen that patients were on at the time. This did not consider other switches during their duration on treatment. This is, however, unlikely to have affected the findings as most of the associations found, resonate with those already established in literature. Secondly, the use of an established regimen made it impossible to assess the effect of individual drugs. The conclusions are therefore made by deduction, based on the higher odds of diabetes for some but not for others on a different drug combination. Lastly, the study ignored the biological or metabolic causes of diabetes due to the nature of the design. This was, however, not the aim of the study, as the study aimed to prove the hypothesis of a higher association between ARVs and type-2 DM and this has been successfully established.

More prospective research needs to be ongoing in the HIV/AIDS arena to find the alternative drugs that are safe for use. Such studies should include but not limited to studies which aim to confirm the risk of cARVs on incident type-2 diabetes, the mechanism through which these drugs cause type-2 DM, the biological factors that could predict the future development of diabetes in individuals and populations, and possible drugs that could counter the diabetogenic effects of the identified drugs without reducing their potency as ARVs. Regular monitoring of patients on cARVs is crucial in order to control the long-term effects and complications of type-2 DM in the HIV/AIDS context.

## Conclusion

This study has shed light on the association between different ARV regimens and type-2 DM. Furthermore, not only was the associated ARV regimen identified but the probable drugs associated with type-2 DM were also identified. Other predictors of type-2 DM included a longer duration on cARVs. ARVs are important for survival in PLWHIV, but it’s also important to ensure a good quality of life for such patients. It is therefore important to continuously monitor such patients, avoid the use of drugs that are likely to cause diabetes and prepare health services for the possible increase of diabetic cases among PLWHIV.

## Supporting information

S1 Data (DTA)
